The article "Dissecting the role of novel EZH2 inhibitors in primary glioblastoma cell cultures: effects on proliferation, epithelial-mesenchymal transition, migration, and on the pro-inflammatory phenotype" was retracted in 2023. Reasons: duplicated images; overlap with earlier publications; unreliable data; concerns about the data.

# Dissecting the role of novel EZH2 inhibitors in primary glioblastoma cell cultures: effects on proliferation, epithelial-mesenchymal transition, migration, and on the pro-inflammatory phenotype

**DOI:** 10.1186/s13148-019-0763-5

**Published:** 2019-12-02

**Authors:** Giulia Stazi, Ludovica Taglieri, Alice Nicolai, Annalisa Romanelli, Rossella Fioravanti, Stefania Morrone, Manuela Sabatino, Rino Ragno, Samanta Taurone, Marcella Nebbioso, Raffaella Carletti, Marco Artico, Sergio Valente, Susanna Scarpa, Antonello Mai

**Affiliations:** 1 Department of Chemistry and Technologies of Drugs, Sapienza University of Rome, P.le A. Moro 5, 00185 Rome, Italy; 2 Department of Experimental Medicine, Sapienza University of Rome, P.le A. Moro 5, 00185 Rome, Italy; 3 Alchemical Dynamics s.r.l, 00125 Roma, Italy; 4 Department of Sense Organs, Sapienza University of Rome, P.le A. Moro 5, 00185 Rome, Italy; 5 Department of Radiologic, Oncological, and Anatomical and Pathological Sciences, Sapienza University of Rome, P.le A. Moro 5, 00185 Rome, Italy

**Keywords:** Epigenetics, EZH2, Histone methylation, Glioblastoma, EMT, Inflammation

## Abstract

**Background:**

Glioblastoma (GBM) is the most lethal and aggressive malignant primary brain tumor in adults. After surgical resection of the tumor, the patient typically should be subjected to chemotherapy (temozolomide, TMZ) and concomitant radiotherapy. Since the TMZ treatment does not lead to complete remission and often develops resistance, the identification of efficacious therapeutics is strongly to pursue. Among the epigenetic players, the H3K27 methyltransferase (MT) EZH2 (enhancer of zeste homologue 2) has been found overexpressed or mutated in several human cancers including gliomas, and its overexpression is associated with poor outcome in GBM. Two EZH2 inhibitors (EZH2i), UNC1999 and GSK343, suppressed GBM growth in vitro and in vivo indicating that EZH2i can be potential drugs against GBM.

**Results:**

Two new EZH2i, MC4040 and MC4041, were designed, prepared, and tested by us to determine their effects in primary GBM cell cultures. MC4040 and MC4041 displayed single-digit micromolar inhibition of EZH2, 10-fold less potency against EZH1, and no activity towards other MTs. In primary GBM cells as well as in U-87 GBM cells, the two compounds reduced H3K27me3 levels, and dose- and time-dependently impaired GBM cell viability without inducing apoptosis and arresting the cell cycle in the G0/G1 phase, with increased p21 and p27 levels. In combination with TMZ, MC4040 and MC4041 displayed stronger, but not additive, effects on cell viability. The potent clinical candidate as EZH2i tazemetostat, alone or in combination with TMZ, exhibited a similar potency of inhibition of GBM cell growth when compared to MC4040 and MC4041. At the molecular level, MC4040 and MC4041 reduced the VEGFR1/VEGF expression, reversed the epithelial-mesenchymal transition (EMT), and hampered cell migration and invasion attenuating the cancer malignant phenotype. Treatment of GBM cells with MC4040 and MC4041 also impaired the GBM pro-inflammatory phenotype, with a significant decrease of TGF-β, TNF-α, and IL-6, joined to an increase of the anti-inflammatory cytokine IL-10.

**Conclusions:**

The two novel EZH2i MC4040 and MC4041 impaired primary GBM cell viability, showing even stronger effects in combination with TMZ. They also weakened the aggressive malignant phenotype by reducing angiogenesis, EMT, cell migration/invasion and inflammation, thus they may be considered potential candidates against GBM also for combination therapies.

## Introduction

Glioblastoma (GBM) is the most common and aggressive malignant primary brain tumour in adults [1]. The standard treatment consists of surgical resection of the tumour, followed by chemotherapy and concomitant radiotherapy [2]. To date, the sole drug in use against GBM is the alkylating agent temozolomide (TMZ). Despite such combined and articulated regimen, the current therapeutic strategy is not a cure, and the prognosis for GBM patients remains poor with a median survival around 15 months and a 2-year survival rate of about 27%. Additionally, the intrinsic or acquired resistance to TMZ reduces the therapeutic success. Several different factors obstacle the development of successful treatments against GBM, including its intrinsic aggressive and infiltrative nature, and the high inter- and intra-tumour variability at the histopathological, genetic and epigenetic levels [3, 4]. Therefore, alternative and/or complementary therapeutic targets and strategies need to be found. In the last years, efforts have been done to this aim, and researchers started also to evaluate the possibility to use immunotherapy; however, no success has been yet recorded [5]. A growing number of literature evidences prove that epigenetic mechanisms are implied in the development and progression of GBM [6–8]. The *S*-adenosyl-l-methionine (SAM)-dependent methyltransferase EZH2 (enhancer of zeste homologue 2) is the catalytic subunit of the polycomb repressive complex 2 (PRC2), responsible of the methylation of the lysine 27 of the histone 3 (H3K27), a mark of gene silencing [9]. EZH2 and the PRC2 complex can silence many genes involved in cell proliferation, cell-cycle regulation, cell differentiation, and self-renewal [9]. EZH2 has been found overexpressed or mutated in several human cancers [9] including gliomas, where its overexpression has been correlated with the glioma grade and poor prognosis [10, 11]. Accordingly, EZH2 depletion by RNA interference in glioma cells led to cell growth inhibition and cycle arrest in the G0/G1 phase both in vitro and in vivo [10, 12]. Moreover, EZH2 regulates cell stemness and epithelial to mesenchymal transition (EMT) in gliomas [11], and it is involved in the development of multidrug resistance, with its inhibition restoring the normal drug sensitivity in GBM [13].

To date, numerous molecules have been synthesized and evaluated in preclinical and clinical settings as competitive, catalytic EZH2 inhibitors (Fig. 1) [14], and some of them including GSK126, tazemetostat and CPI-1205, are being tested in clinical studies [14]. Moreover, few of them (UNC1999 and GSK343, an analogue of GSK126) have been tested against GBM *in vitro* and *in vivo*, proving the relevance of EZH2 as target to fight in this disorder [15, 16].

**Fig. 1:** Structures of EZH2 inhibitors studied in a clinical setting and/or in GBM models, including MC4040 and MC4041 used in the present research

Recently, through a pruning strategy applied on known indazole-containing EZH2 inhibitors (EZH2i) (such as EPZ005687 and UNC1999, Fig. 1), our group reported the novel pyrazole-based EZH2i MC3629 (Fig. 1), potent at low micromolar doses and able to reduce H3K27me3 levels, to arrest cell proliferation and to induce autophagy in a panel of cancer cell lines (SK-N-BE neuroblastoma, MDA-MB231 breast cancer, and K562 leukaemia cells) [17]. When tested in Sonic Hedgehog (SHH) medulloblastoma (MB) stem-like cells, MC3629 impaired cell proliferation and self-renewal inducing apoptosis [18]. In MB xenografted mice, MC3629 showed a significant decrease of tumour volume, a reduction of stemness and cell proliferation, and induction of apoptosis [18]. Mimicking the benzo-cracking approach followed for MC3629, starting from the structures of known indole-based EZH2 inhibitors (such as GSK126, EI1, and CPI-1205, Fig. 1) we designed and synthesized a series of pyrrole dimethylpyridone-containing compounds to be tested against EZH2. Among them, MC4040 and MC4041 (Fig. 1) were tested in GBM cells including primary GBM cell cultures, to determine their antiproliferative effects alone and in combination with temozolomide. To dissect the molecular mechanisms of these new EZH2 inhibitors, their efficacy in mitigating the GBM malignant phenotype has been determined through the reduction of VEGFR1/VEGF expression, reversion of the EMT process, inhibition of invasive phenotype, and decrease of inflammatory cytokines levels.

## Materials and Methods

### Chemistry

Melting points were determined on a Buchi 530 melting point apparatus and are uncorrected. 1H NMR (nuclear magnetic resonance) spectra were recorded at 400 MHz on a Bruker AC 400 spectrometer; chemical shifts are reported in δ (ppm) units relative to the internal reference tetramethylsilane (Me_4_Si). EIMS spectra were recorded with a Fisons Trio 1000 spectrometer; only molecular ions (M+) and base peaks are given. All compounds were routinely checked by TLC (thin layer chromatography), 1H NMR and 13C NMR spectra. TLC was performed on aluminium-backed silica gel plates (Merck DC, Alufolien Kieselgel 60 F254) with spots visualized by UV light. All solvents were reagent grade and, when necessary, were purified and dried by standard methods. The concentration of solutions after reactions and extractions involved the use of a rotary evaporator operating at reduced pressure of ca. 20 Torr. Organic solutions were dried over anhydrous sodium sulphate. Elemental analysis has been used to determine the purity of the described compounds, that is > 95%. Analytical results are within ± 0.40% of the theoretical values. All chemicals were purchased from Sigma-Aldrich Chimica, Milan (Italy), or from Alfa Aesar, Karlsruhe (Germany), and were of the highest purity.

### Synthesis of 1-(3-bromophenyl)-2,5-dimethyl-1H-pyrrole (1)

A solution of 2,5-hexanedione (8.50 mmol, 1.2 eq, 1 mL) in glacial acetic acid (3 mL) was prepared in a flame dried sealed tube, and 3-bromoaniline (7.08 mmol, 1.0 eq, 1.22 g, 0.77 mL) was added to the solution. The reaction solution was stirred at 100 °C for 2 h. After this time the reaction was complete, the acetic acid was removed in vacuo (azeotrope with toluene) and the residue was purified by silica gel chromatography, eluting with the *n*-hexane:chloroform (60:1) mixture. The product was obtained as a white solid (5.31 mmol, 1.33 g, 75%). m.p. 84–85 °C (*n*-hexane). ^1^H-NMR (CDCl_3_, 400 MHz, δ; ppm): δ_H_ 1.96 (6H, s, C(2)CH_3_, C(5)CH_3_), 5.82 (2H, s, C(3)H, C(4)H pyrrole), 7.08–7.11 (1H, ddd, *J* = 7.6 Hz, 1.8 Hz, 0.8 Hz, aromatic proton), 7.26 (1H, t, *J* = 8 Hz, aromatic proton), 7.32 (1H, t, *J* = 1.6 Hz, aromatic proton), 7.45-7.48 (1H, ddd, *J* = 8 Hz, 1.8, 1.2 Hz, aromatic proton) ppm. MS (EI) m/z [M]^+^: 249.02. The reported data are in good agreement with the literature [19, 20].

### General procedure for the synthesis of the intermediates 2a,b. Example: Synthesis of 1-(3-(2,5-dimethyl-1H-pyrrol-1-yl)phenyl)piperidine (2b)

In a flame dried sealed tube, 1-(3-bromophenyl)-2,5-dimethyl-1*H*-pyrrole **1** (1.59 mmol, 1.0 eq, 0.40 g), piperidine (3.20 mmol, 2 eq, 0.27 g, 0.316 mL), palladium(II) acetate (Pd(OAc)_2_) (0.024 mmol, 1.5% mol, 5.4 mg), tri-*tert*-butylphosphonium tetrafluoroborate (PH(tBu)_3_BF_4_) (0.0192 mmol, 1.2% mol, 5.6 mg), and potassium *tert*-butoxide (3.59 mmol, 2.25 eq, 0.404 g) were added in sequence and suspended in dry toluene (3.0 mL). The system was degassed (N_2_) and left under stirring at 80 °C for 16 h. After this time, the reaction was quenched by adding ethyl acetate, and it was filtered over celite pad. The filtrate was concentrated in vacuo and the crude was purified by silica gel chromatography eluting with the *n*-hexane:ethyl acetate (5:1) mixture, to give the 1-(3-(2,5-dimethyl-1*H*-pyrrol-1-yl)phenyl)piperidine **2b** as a colourless oil (1.27 mmol, 0.32 g, 80%). ^1^H-NMR (*d*_*6*_-DMSO, 400 MHz, δ; ppm): δ_H_ 1.59-1.60 (6H, m, piperidine protons), 1.97 (6H, s, C(2)CH_3_, C(5)CH_3_ pyrrole), 3.17-3.20 (4H, m, piperidine protons), 5.70 (2H, s, C(3)H, C(4)H pyrrole), 6.56 (1H, dd, *J* = 7.6 Hz, 2.0 Hz, aromatic proton), 6.69 (1H, t, *J* = 2.0 Hz, aromatic proton), 6.97 (1H, dd, *J* = 7.6 Hz, 2.0 Hz, aromatic proton), 7.29 (1H, t, *J* = 7.6 Hz, aromatic proton) ppm. MS (EI) m/z [M]^+^: 254.18.

### Chemical and physical characterization of 4-(3-(2,5-dimethyl-1H-pyrrol-1-yl)phenyl)morpholine (2a): light yellow oil (yield 82%)

^1^H-NMR (d_6_-DMSO, 400 MHz, δ; ppm): δ_H_ 1.97 (6H, s, C(2)CH_3_, C(5)CH_3_ pyrrole), 3.16 (4H, t, J = 11.0 Hz, morpholine protons), 3.73 (4H, t, J = 11.0 Hz, morpholine protons), 5.76 (2H, s, C(3)H, C(4)H pyrrole), 6.63 (1H, dd, J = 8.2 Hz, 2.0 Hz, aromatic proton), 6.73 (1H, t, J = 2.0 Hz, aromatic proton), 6.99 (1H, dd, J = 8.2 Hz, 2.0 Hz, aromatic proton), 7.32 (1H, t, J = 8.0 Hz, aromatic proton) ppm. MS (EI) m/z [M]^+^: 256.16.

### General procedure for the synthesis of pyrrole-3-carboxylic acids (3a,b). Example: Synthesis of 2,5-dimethyl-1-(3-morpholinophenyl)-1H-pyrrole-3-carboxylic acid (3a)

In a sealed tube, 4-(3-(2,5-dimethyl-1*H*-pyrrol-1-yl)phenyl)morpholine **2a** (0.84 mmol, 1.0 eq, 0.22 g) was dissolved in 1,2-dichloroethane (2 mL), the solution was cooled to 0 °C, and trichloroacetyl chloride (2.53 mmol, 3.0 eq, 0.28 mL) was added dropwise to the solution. The reaction was stirred at 70 °C for 1 h. After this time the reaction was complete, and the volatiles were removed in vacuo. The residue was dissolved in an ethanol/tetrahydrofuran (1:1) mixture, the solution was cooled to 0 °C, and 2 M aqueous solution of potassium hydroxide (8.43 mmol, 10 eq, 0.47 g) was added dropwise to the solution. The reaction mixture was stirred at room temperature for 1 h and then at 80 °C for 3 h. After this time the reaction was complete, and the organic solvents were removed in vacuo. The byproducts were extracted from the basic aqueous layer with ethyl acetate (3 × 10 mL). The aqueous layer was then cooled to 0 °C and acidified till pH 2 by addition of a 2 M aqueous solution of HCl. The product precipitated, and it was filtered, rinsed with distilled water and dried in oven (60 °C). Yield 69%. m.p. 173–175 °C (toluene/acetonitrile). ^1^H-NMR (*d*_*6*_-DMSO, 400 MHz, δ; ppm): δ_H_ 1.94 (3H, s, C(5)CH_3_ pyrrole), 2.23 (3H, s, C(2)CH_3_ pyrrole), 3.15-3.18 (4H, m, morpholine protons), 3.71–3.74 (4H, m, morpholine protons), 6.21 (1H, s, C(4)H pyrrole), 6.76 (1H, s, aromatic proton), 7.02 (1H, d, *J* = 7.6 Hz, aromatic proton), 7.13 ( 1H, d, *J* = 7.6 Hz, aromatic proton), 7.41 (1H, t, *J* = 7.6 Hz, aromatic proton), 11.66 (1H, bs, COO*H*) ppm. MS (EI) m/z [M]^+^: 300.15.

### Chemical and physical properties of 2,5-dimethyl-1-(3-(piperidin-1-yl)phenyl)-1H-pyrrole-3-carboxylic acid (3b): m.p. 178–180 °C (toluene/acetonitrile)

^1^H-NMR (*d*_*6*_-DMSO, 400 MHz, δ; ppm): δ_H_ 1.56 (6H, m, piperidine protons), 1.94 (3H, s, C(5)CH_3_ pyrrole), 2.21 (3H, s, C(2)CH_3_ pyrrole), 3.19-3.21 (4H, m, piperidine protons), 6.20 (1H, s, C(4)H pyrrole), 6.59 (1H, d, *J* = 7.6 Hz, aromatic proton), 6.75 (1H, bs, aromatic proton), 7.30 (1H, dd, *J* = 8 Hz, 2 Hz, aromatic proton), 7.33 (1H, t, *J* = 8 Hz, aromatic proton), 11.56 (1H, bs, COO*H*) ppm. MS (EI) m/z [M]^+^: 298.17.

### General procedure for the synthesis of pyrrole amides (MC4040 and MC4041). Example: Synthesis of N-((4,6-dimethyl-2-oxo-1,2-dihydropyridin-3-yl)methyl)-2,5-dimethyl-1-(3-morpholinophenyl)-1H-pyrrole-3-carboxamide (MC4040)

In a flame dried round bottom flask, 2,5-dimethyl-1-(3-morpholinophenyl)-1*H*-pyrrole-3-carboxylic acid (0.33 mmol, 1.0 eq, 100.0 mg) was solved in dry *N*,*N*-dimethylformamide (DMF) (1 mL) under N_2_ atmosphere. Triethylamine (2.33 mmol, 7.0 eq, 0.24 mL), and *O*-(benzotriazol-1-yl)-*N,N,N’,N’*-tetramethyluronium tetrafluoroborate (TBTU) (0.40 mmol, 1.2 eq, 0.13 g) were added to the reaction solution, and the system was left under stirring at room temperature for 40 min. After this time, 3-(aminomethyl)-4,6-dimethylpyridin-2(1*H*)-one hydrochloride **4** [21] (0.37 mmol, 1.1 eq, 69 mg) was added to the solution and the reaction was stirred under N_2_ at 60 °C for 4 h. After this time, the reaction was complete, and it was quenched by addition of 3 mL of a saturated aqueous solution of NaCl. The product precipitated, and it was filtered and rinsed with distilled water. The solid was dried and further purified by silica gel chromatography eluting with the chloroform:methanol (35:1) mixture, to give MC4040 (0.18 mmol, 76.7 mg, 53%). m.p. 178-180 °C (acetonitrile). ^1^H NMR (DMSO-*d*_*6*_, 400 MHz, δ, ppm): δ_H_ 1.92 (3H, s, C(5)C*H*_3_ pyrrole), 2.12 (3H, s, C*H*_3_ dimethylpyridone), 2.18 (3H, s, C*H*_3_ dimethylpyridone), 2.21 (3H, s, C(2)C*H*_3_ pyrrole), 3.16 (4H, t, *J* = 4.6 Hz, morpholine protons), 3.72 (4H, t, *J* = 4.6 Hz, morpholine protons), 4.22 (2H, d, *J* = 5.2 Hz, -C*H*_2_NHCO-), 5.86 (1H, s, dimethylpyridone C*H*), 6.26 (1H, s, C(4)*H* pyrrole), 6.64 (1H, d, *J* = 8 Hz, aromatic proton), 6.76 (1H, s, aromatic proton), 7.03 (1H, d, *J* = 7.2 Hz, aromatic proton), 7.34-7.39 (2H, m, aromatic proton and -CH_2_N*H*CO-), 11.47 (1H,bs, -NH- pyridone) ppm. MS (EI) m/z [M]^+^: 434.23.

### Chemical and physical characterization of N-((4,6-dimethyl-2-oxo-1,2-dihydropyridin-3-yl)methyl)-2,5-dimethyl-1-(3-(piperidin-1-yl)phenyl)-1H-pyrrole-3-carboxamide (MC4041)

^1^H NMR (DMSO-*d*_*6*_, 400 MHz, δ, ppm): δ_H_ 1.54–1.60 (6H, m, piperidine protons), 1.92 (3H, s, C(5)C*H*_3_ pyrrole), 2.11 (3H, s, C*H*_3_ dimethylpyridone), 2.18 (3H, s, C*H*_3_ dimethylpyridone), 2.21 (3H, s, C(2)C*H*_3_ pyrrole), 3.18–3.20 (4H, m, piperidine protons), 4.22 (2H, d, *J* = 5.2 Hz, -C*H*_2_NHCO-), 5.86(1H, s, dimethylpyridone C*H*), 6.25 (1H, s, C(4)H pyrrole), 6.55 (1H, d, *J* = 7.6 Hz, aromatic proton), 6.70 (1H, bs, aromatic proton), 7.01 (1H, dd, *J* = 2 Hz, 8.4 Hz, aromatic proton), 7.34 (1H, t, *J* = 8 Hz, aromatic proton), 7.40 (1H, t, *J* = 5.2 Hz, -CH_2_N*H*CO-), 11.48 (1H, bs, -NH- pyridone). m.p. 135-137 °C (benzene); Yield = 55%. MS (EI) m/z [M]^+^: 432.25.

### Biochemistry

#### EZH2/PRC2 complex assay

The EZH2 substrate (0.05 mg/mL core histone) was added in the freshly prepared reaction buffer (50 mM Tris-HCl (pH 8.0), 50 mM NaCl, 1 mM EDTA, 1 mM DTT, 1 mM PMSF, 1% DMSO). The PRC2 complex [complex of human EZH2, human EED, human SUZ12, human AEBP2, and human RbAp48] was delivered into the substrate solution and the mixture was mixed gently. Afterwards, the tested compounds dissolved in DMSO were delivered into the enzyme/substrate reaction mixture by using Acoustic Technology (Echo 550, LabCyte Inc. Sunnyvale, CA) in a nanolitre range, and ^3^H-SAM was added into the reaction mixture to initiate the reaction. The reaction mixture was incubated for 1 h at 30 °C and then it was delivered to filter-paper for detection. The data were analysed using Excel and GraphPad Prism software for IC_50_ curve fits.

#### EZH1/PRC2 complex, G9a, PRMT1, and DNMT1 assays

The appropriate methyltransferase (MT) substrate (0.05 mg/ml core histone for EZH1 complex, 5 μM histone H3 (1-21) peptide for G9a, 5 μM histone H4 for PRMT1, and 0.001 mg/ mL poly(dI-dC) for DNMT1) was added in freshly prepared reaction buffer (50 mM Tris-HCl (pH 8.5), 5 mM MgCl_2_, 50 mM NaCl, 0.01 % Brij35, 1 mM DTT, 1 % DMSO). The MT enzyme was delivered into the substrate solution and the mixture was mixed gently. Afterwards, the tested compounds dissolved in DMSO were delivered into the enzyme/substrate reaction mixture by using Acoustic Technology (Echo 550, LabCyte Inc. Sunnyvale, CA) in nanolitre range, and 1 μM ^3^H-SAM was also added into the reaction mixture to initiate the reaction. The reaction mixture was incubated for 1 h at 30 °C and then it was delivered to filter-paper for detection. The data were analysed using Excel and GraphPad Prism software for IC_50_ curve fits.

### Molecular modelling

Molecular docking simulations were run on MC4041 and MC4040 modelled conformation to gather information on their likely binding modes into EZH2. To this, eight experimental structures of human PRC2 in complex with several inhibitors (pdb entry codes: 4w2r, 5ch2, 5ij7, 5ls6, 5ch1, 5hyn, 5ij8 and 6b3w) were retrieved from PDB [22] (www.rcsb.org). PCR2 co-crystallized complexes were structurally inspected and experimentally missing residues were modelled by means of the programme MODELLER ver 9.19 [23]. To avoid insertion of too unfolded parts, only 10 of the about 80 initial missing residues were fully modelled. The internal gaps were all automatically filled similarly as described in the MODELLER manual. The modelled complexes were then subjected to single-point energy geometry optimization in explicit water and the minimized complexes. Cross-docking experiments were performed with the programme PLANTS [24] using the ChemPlp scoring functions. Chemical compounds were parametrized with AM1-BCC [25] partial charges and GAFF v2.1 [26] Lennard-Jones and valence parameters, using AmberTools 17 antechamber and parmchk2 utilities [27, 28]. The OPC [29] water model and AMBER14SB [30] forcefield were used during complexes minimizations. By means of molecular mechanics/generalized Born surface area (MMGBSA) method [31], the protein-ligand binding free energies were evaluated. MarvinSketch 17.1.16 (http://www.chemaxon.com) was used for drawing the chemical structures, which were then converted in 3D-Structures with OpenBabel 2.4.1 [32] employing MMFF94 [33] force field.

### In cell studies

#### Cell culture and treatments

Three human GBM primary cell cultures (GL1, GL2, GL3) were established from surgical tissues of three different patients, and in addition, one human normal dermal fibroblast primary culture (HF) was obtained. All the primary cell cultures were prepared as previously described [34]. Additionally, a human GBM cell line U-87 MG (ATCC HTB-14), here indicated as U-87, was utilized. The U-87 cell line was grown in EMEM medium supplemented with 10% foetal calf serum (FCS), 2 mM glutamine, 50 U/mL penicillin-streptomycin, 1 mM non-essential amino acid, 1 mM sodium pyruvate. GL1, GL2, GL3 and HF were grown in DMEM medium supplemented with 10% FCS, 2 mM glutamine, 50 U/mL penicillin-streptomycin. MC 4040 and MC 4041 were solubilized in dimethylsulfoxide (DMSO) (Sigma-Aldrich) at 10 mM stock solution and utilized to final concentrations from 10 to 50 μM. Control cells were treated with equivalent amounts of DMSO in each experiment. Staurosporine (Sigma-Aldrich) was dissolved in DMSO in a 1 mM stock solution and used at 5 μM for 6 h. Tazemetostat was solubilized in a 10 mM DMSO stock solution and utilized at 25 μM. Temozolomide was solubilized in a 100 mM DMSO stock solution and utilized at 100 μM.

#### Cytotoxicity assay

To determine cytotoxicity, sulforhodamine B colorimetric assay was performed: 1.5 × 10^4^ cells were plated on 96 well plates, grown for 24 h and treated with different concentrations of MC4040 and MC4041 (10, 25, and 50 μM), with tazemetostat (25 M) and/or with temozolomide (100 μM) for 48, 72, 96 and 120 h. Control cells were treated with equivalent amounts of DMSO. Cells were then fixed with 50% trichloroacetic acid for 1 h at 4 °C and stained for 30 min at room temperature with 0.4% sulforhodamine B in 1% acetic acid. Excess dye was removed by washing four times with 1% acetic acid. Protein-bound dye was dissolved in 10 mM TRIS pH 10, and optical density (OD) was determined at 510 nm using a microplate reader.

#### Flow cytometry analysis

GL1 and U-87 cells were seeded in 60-mm culture plates and grown for 48 h untreated or treated with 25 μM MC4040 and MC4041. The cells were harvested by trypsinization, washed twice with cold PBS, and fixed in 70% ethanol at 4 °C overnight. After fixation, the cells were rinsed with PBS and incubated with 10 mg/mL RNase and 1 mg/mL propidium iodide (Sigma-Aldrich) at room temperature for 2 h in the dark. The cell cycle distribution was measured and analysed by FACS Calibur flow cytometry using the Cell Quest analysis programme to detect the distribution of subpopulations through the cell cycle. Each experiment was performed in triplicate.

### Western blot analysis

Cell lysates were obtained scraping the cells in lysis buffer 1% Triton, 0.1% SDS, 150 mM NaCl, 50 mM TRIS-HCl pH 7.4, 2 mM EDTA plus protease inhibitor cocktail tablet (Roche Applied Sciences) for 30 min at 4 °C. The lysates were then centrifuged at 12,000 rpm for 15 min at 4 °C. The protein concentration was evaluated by Bio-Rad Protein Concentration Assay. Samples of lysate (100 μg) were separated by molecular weight on 10 or 12% SDS-PAGE and then transferred into a nitrocellulose membrane. Blots were blocked for 1 h at room temperature in 5% non-fat dry milk and then incubated overnight at 4 °C with rabbit polyclonal anti-H3K27me3 antibodies (cell signalling technology) diluted 1:1000 in 5% BSA, 0.1% Tween 20 TRIS-buffered saline, or alternatively for 1 h at room temperature with all the other primary antibodies in TRIS-buffered saline. The primary antibodies were the following: mouse anti-Parp1 (1:500 diluted) (Santa Cruz Biotechnology); rabbit anti-p21 Waf1/Cip1 (1:1000 diluted) (Cell Signaling); mouse anti-p27 (1:500 diluted) (Santa Cruz Biotechnology); rabbit anti-ß-actin (1:1000 diluted) (Sigma-Aldrich) rabbit anti-E-cadherin (1:1000 diluted) (Gene Tex); rabbit anti-N-cadherin (1:1000 diluted) (Gene Tex); rabbit anti-MMP-2 (1:1000 diluted) (Gene Tex); rabbit anti-MMP-9 (1:500 diluted) (Biomol); mouse anti-TGF-ß (1:500 diluted) (Santa Cruz Biotechnology); rabbit anti-TNF-α (1:1000 diluted) (Elabscience); mouse anti-IL-6 (1:500 diluted) (Santa Cruz Biotechnology); mouse anti-IL-10 (1:500) (Santa Cruz Biotechnology). Blots were washed in TRIS-buffered saline with 0.1% Tween 20 and then incubated with horseradish peroxidase-conjugated anti-rabbit or anti-mouse antibodies (1:5000 diluted) (Sigma-Aldrich). The filters were then developed by enhanced chemiluminescence (Super Signal West Pico Chemiluminescent Substrate, Thermo Scientific) using Kodak X-Omat films. The densitometry quantitation of the bands was performed using Image J software.

### Immunofluorescence

The cells were grown directly on Labteck chamber slides (Nunc) for 24 h and then used untreated or treated for 48 h with 25 μM MC4040 or MC4041. The cells were then washed with PBS with Ca/Mg and fixed with absolute cold methanol for 5 min (only for nestin staining) or with 4% buffered paraformaldehyde for 20 min at 4 °C (for all other antibodies). The cells were incubated with 3% bovine serum albumin for 1 h at room temperature and then with anti-glial fibrillary acidic protein (GFAP) rabbit antibody (1:200 diluted, Abcam) or anti-vascular endothelial growth factor (VEGF) mouse antibody (1:100 diluted, Santa Cruz Biotechnology) or anti-VEGF-receptor1 (VEGFR1) mouse antibody (1:100 diluted, Abcam) for 1 h at room temperature; with anti-nestin rabbit antibody (1:200 diluted, Abcam) overnight at 4 °C. Cells were then washed twice with PBS with Ca/Mg and then incubated with the secondary anti-rabbit antibody Alexa Fluor 594 conjugated (Invitrogen, 1:400 diluted) or anti-mouse antibody Alexa Fluor 488 conjugated (Invitrogen, 1:200 diluted) for 1 h at room temperature. The cells were finally washed twice with PBS with Ca/Mg, mounted with Prolong Antifade reagent (Life Technologies) and analysed by a fluorescence microscope (Olympus BX52); imagine acquisition and processing were conducted by IAS 2000 software.

### Invasion assay

Invasion assay was performed with Bio Coat Matrigel Invasion Chambers (Corning), consisting of inserts with an 8 μm pores size membrane that was previously treated with Matrigel matrix. For invasion assay 2.5 × 10^5^/mL cells were plated in serum-free medium plus vehicle DMSO or in serum-free medium plus 20 μM MC4040 and MC4041 in the insert chamber, the lower chamber instead contained only complete medium (with FCS). After 48 h of culture at standard conditions, the inserts were washed with PBS with Ca/Mg and fixed by 100% methanol for 20 min at 4 °C, then washed twice with PBS with Ca/Mg and stained for 20 min at room temperature with crystal violet. The inserts were then mounted on a slide with glycerol and the cells that migrated through the filter pores to the lower side of the membrane were counted by an optical microscope (Olympus BX52). Imagine acquisition and processing were conducted by IAS 2000 software.

### Statistical analysis and graphic programmes

All results were analysed by ANOVA, and the significance was evaluated by the Tukey HSD post hoc test (Honestly Significant Difference). All figures were elaborated with Adobe Photoshop CS5 and all graphs with Graph Pad Prism 5.0

## Results

### Synthesis of MC4040 and MC4041

The synthesis of MC4040 and MC4041 started with the preparation of the pyrrole key intermediate **1** through a Paal-Knorr reaction (Scheme 1). More in detail, 2,5-hexanedione was treated with 3-bromoaniline in the presence of acetic acid to afford the 1-(3-bromophenyl)-2,5-dimethyl-1*H*-pyrrole **1**, which underwent a Buchwald-Hartwig reaction by using morpholine or piperidine, palladium (II) acetate (Pd(OAc)_2_) as catalyst and tri-*tert*-butylphosphonium tetrafluoroborate (PH(tBu)_3_BF_4_) as ligand, and providing **2a** and **2b**, respectively, in good yields (Scheme 1) [35]. The subsequent Friedel-Craft acylation performed on **2a,b** with trichloroacetyl chloride gave the corresponding crude 3-trichloroacetyl pyrroles, which were directly converted into the related 3-pyrrolecarboxylic acids **3a,b** (Scheme 1). Further coupling of the acids **3a,b**, activated with *O*-(benzotriazole-1-yl)-*N,N,N’,N’*-tetramethyluronium tetrafluoroborate (TBTU), with the 3-(aminomethyl)-4,6-dimethylpyridin-2(1*H*)-one hydrochloride **4** [21] in the presence of triethylamine yielded the final compounds MC4040 and MC4041 (Scheme 1).

**Scheme 1:** Reagents and conditions: (a) glacial acetic acid, sealed tube, 100 °C, 1.5 h (35-80%); (b) Pd(OAc)_2_, PH(tBu)_3_BF_3_, potassium *tert*-butoxide, dry toluene, sealed tube, N_2_, 80 °C, 4 h (76-80%); (c) trichloroacetyl chloride, dry 1,2-dichloroethane, sealed tube, 0 °C to 70 °C, 1 h; (d) I. 2 N KOH (aq), EtOH, r.t. to 60 °C; II. 2 N HCl (aq) (54-73 %); (e) triethylamine, TBTU, dry DMF, N_2_, r. t., 4 h (52-75%)

### Assessment of EZH2 inhibition activity and selectivity against other methyltransferases

The newly synthesized compounds have been screened in a 10-dose IC_50_ mode with 2-fold serial dilution starting from 200 μM solutions, in an in vitro enzymatic assay against a human five component PRC2 complex, containing EZH2, EED, SUZ12, RbAp48, and AEBP2, to evaluate their ability to inhibit the EZH2 catalytic activity. The assay was performed using core histone as substrate and ^3^H-SAM as co-substrate. *S*-Adenosyl-l-homocysteine (SAH), GSK126 and tazemetostat were used as reference compounds. Compounds MC4040 and MC4041 proved to inhibit EZH2 displaying IC_50_ values in the low micromolar range (Table 1). Both compounds proved to inhibit also the PRC2-EZH1 complex in vitro, displaying however 10-fold higher IC_50_ values (Table 1). When tested against other SAM-dependent methyltransferases such as G9a (another lysine methyltransferase), PRMT1 (an arginine methyltransferase), and DNMT1 (a DNA methyltransferase), no inhibition was recorded for both compounds up to 200 μM. Only MC4041 showed a slight PRMT1 inhibition (11.9%) at 200 μM.

**Table 1:** IC_50_ values, or percentage of inhibition at 200 μM, of MC4040 and MC4041 against a panel of methyltransferases

Compound	IC_50_, μM^*a*^ or % inhibition at 200 μM				
	EZH2	EZH1	G9a	PRMT1	DNMT1
MC4040	4.06	42.7	NA^*b*^	NA	NA
MC4041	1.06	10.6	NA	11.9%	NA
SAH	34.7				
GSK126	0.009				
TAZ^*c*^	<0.005				

^*a*^Performed in a 10-dose IC_50_ mode with 2-fold serial dilution starting from 200 μM. ^*b*^*NA*, not active. ^*c*^*TAZ*, tazemetostat

### Molecular modelling studies

Molecular modelling studies were performed to highlight any difference in the binding mode of the two novel compounds. Cross-docking experiment revealed that the programme PLANTS is suitable to perform docking experiments for potential ligands on PRC2 as a docking accuracy of 90% was achieved [36]. MC4040 and MC4041 lowest energy docking conformations were associated with the PRC2 protein obtained from the 6b3w complex. Visual inspection of MC4040 and MC4041 docked conformations revealed that although structurally very similar, the two molecules only partially share their binding modes (Fig. 2). In more detail, while the two pyridone and the carboxamide moieties are completely overlapped, the rest of the two molecules assume conformations that tend to gradually separate. In particular, MC4040 and MC4041 pyridone moieties interact with Gly520, Trp51, Phe583, Ala584, Asn585 and Tyr623 residues (Fig. 2), constituting a sub-pocked that lay in the EZH2 SAM binding site (not shown). Hydrogen bonds (not shown) are possible among Gly520 oxygen and the inhibitors’ pyridone NHs (distance O_Gly520_**···**N_inhibitors_ = 2.886 Å) and among Trp521 amidic NH and inhibitors’ pyridone carbonyl oxygens (distance N_Trp521_**···**O_inhibitors_ = 3.029 Å). The central pyrrole-3-carboxamides portions, almost overlapped, also share the same interactions, and are trapped in a rounded hydrophobic cage formed mostly by Ile109, Met110, Tyr111, Phe665, Thr678 and Arg685 side chains (see magenta surfaces in Fig. 2). Regarding the phenylpiperidine and phenylmorpholine portions of MC4040 and MC4041 inhibitors, the docked conformations indicate the MC4040 morpholine group to be stuck in a sub-pocked defined by Ser112, His213, Val657, Thr678, and Arg679. Differently, the piperidine of the MC4041 pose was shifted and buried in a high hydrophobic environment surrounded by His213, Arg236, Tyr658, and Tyr661.

**Fig. 2:** **a** MC4040 (carbon atoms in black) docked conformation into PCR2. Only surface (blue) and names of residues within 5 Å are displayed. Close contact surfaces with the pyridone moiety are coloured in pink. Close contact surfaces with the pyrrole-3-carboxamide central group are coloured in magenta and contact surfaces with the piperidine heterocycle are coloured in yellow. Residue numbering is taken from the 6b3w complex. **b** MC4041 (carbon atoms in dark grey) docked conformation into PCR2. Only surface (blue) and names of residues within 5 Å are displayed. Close contact surfaces with the pyridone moiety are coloured in pink. Close contact surfaces with the pyrrole-3-carboxamide central group are coloured in magenta and contact surfaces with the piperidine heterocycle are coloured in orange. Residue numbering are taken from the 6b3w complex

Although the overall interaction pattern of either MC4040 or MC4041 seem quite similar, the piperidine of compound MC4041 seems to establish a larger number of positive van der Waals interactions, accounting at least in part for its higher EZH2 inhibition potency. By means of molecular mechanics/generalized Born surface area (MMGBSA) method [37], the protein-ligand binding free energies were evaluated for all the minimized complexes (Table 2). Analysis of protein-ligand binding free energies (Table 2) showed that MC4041 binds to EZH2 with a better energetic profile than MC4040, in agreement with the experimental biochemical IC_50_ values.

**Table 2:** MMGBSA calculated binding energies (**Δ**G) for MC4040 and MC4041

Ligand	IC_50_ (μM)	GBSA ΔG (kcal/mol)
MC4040	4.06	-23.0432
MC4041	1.06	-30.4428

### Effects of MC4040 and MC4041 on GBM cell proliferation

At the beginning of our studies, we collected patient-derived GBM cells, establishing three primary cell cultures (GL1, GL2, GL3). First, the homogeneity of the neoplastic phenotype of the three human GBM primary cell cultures was determined. Each culture was characterized by immunofluorescence staining of two typical GBM markers: GFAP and nestin. 100 % of cells from GL1, GL2, and GL3 resulted positive for both markers (Fig. 3).

**Fig. 3:** Immunofluorescence of GL1, GL2 and GL3 for GFAP and for nestin

Afterwards, we investigated the effects of the two novel EZH2 inhibitors on cell viability and replication in all the three GBM primary cultures (GL1, GL2, and GL3) and in the GBM cell line U-87. Additionally, a primary culture of human dermal fibroblasts, HF cells, was used as control of somatic not transformed cells. To this scope, GL1, GL2, GL3, U-87, and HF cells were treated for 24, 48, 72, or 96 h with 10, 25, or 50 μM doses of MC4040 and MC4041, separately. After 24 (data not shown) and 48 h of treatment, no effect or a slight decrease of cell viability was evident at the highest doses with both compounds. For longer incubation times (72 and 96 h), the decrease in cell viability became significant also at 10 μM (Fig. 4). Notably, none of the two inhibitors displayed any significant effect on HF proliferation, even after 96 h of treatment at the highest dose (Fig. 4). Based on these data, all the following experiments were performed using MC4040 and MC4041 at the concentration of 25 μM for 72 h.

**Fig. 4:** Cell viability of untreated (ctr) and MC4040- and MC4041-treated cultures expressed as percentage of alive cells. Treatments were performed at 48 h (black), 72 h (dark grey), and 96 h (light grey). *p < 0.05 and **p < 0.01

### Compounds MC4040 and MC4041 reduce H3K27me3 levels in GBM cells

In order to confirm an effective inhibition of EZH2 by MC4040 and MC4041 in a cellular context, U-87, GL1 and HF were treated with DMSO (ctr), or with MC4040, or with MC4041 (both at 25 μM for 72 h), and the levels of H3K27me3 were analysed by western blot. Interestingly, H3K27me3 basal levels were upregulated in GL1 cells when compared to U-87 cells, while no H3K27me3 was detectable in dermal HF cells, as expected (Fig. 5). MC4040 and MC4041 treatment determined an evident downregulation of H3K27me3 in both GBM U-87 and GL1 cells (Fig. 5a), confirming the inhibitory control exerted by both molecules on EZH2. In a time-course experiment, MC4041 while showing no effect after 24 h treatment, reduced H3K27 trimethylation in a time-dependent manner over 72 h (Fig. 5b).

**Fig. 5:** **a** Western blot of U-87, GL1 and HF treated with DMSO (ctr) or with 25 μM MC4040 and MC4041 for 72 h showing H3K27me3 and β-actin levels. The means from densitometry quantifications of three different experiments normalized to β-actin are indicated below each band. ND, not detectable. **b** Time-course experiment performed treating U-87 and GL1 cells with MC4041 (25 μM) for 24, 48, and 72 h. The levels of H3K27me3 are shown (mean from three different experiments) and have been normalized to β-actin

### MC4040 and MC4041 potentiate the effects of temozolomide on GBM cell proliferation

Temozolomide is the sole chemotherapeutic agent available for GBM treatment. Here, we compared the effects of EZH2 inhibition by MC4040, MC4041, or by the clinically studied inhibitor tazemetostat with those of temozolomide. Therefore, U-87 and GL1 were treated either with MC4040 (25 μM), MC4041 (25 μM), tazemetostat (25 μM), or temozolomide (100 μM) for 72, 96, and 120 h. As shown in Fig. 6, the effect of all the three tested EZH2 inhibitors on cell replication was comparable to the effect obtained with temozolomide at all the tested incubation times in both the GBM cell lines.

**Fig. 6:** Cell viability of U-87 and GL1 untreated (ctr) and treated with 25 μM MC4040 or MC4041 or tazemetostat, and with 100 μM temozolomide as single or combined treatments expressed as percentage of alive cells. Treatments were performed at 72 h (**a**, dark grey), 96 h (**b**, light grey) and 120 h (**c**, white). *p < 0.05 and **p < 0.01 for the comparison between single treatments and untreated cells. ^#^indicates *p* < 0.05 for the comparison between each combined treatment and each single treatment with MC4040 and MC4041. ^§^*p* < 0.05 for the comparison between each combined treatment and the single treatment with temozolomide

To check if EZH2 inhibitors in combination with temozolomide could potentiate its effects, we also performed a combination study with each of the three EZH2i in U-87 and GL-1 cells in the same time range observed for the single drug treatment. Pleasingly, the combination had much stronger, but not additive, effects on cell viability already after 72 h, reaching 60% reduction after 96 and 120 h (Fig. 6). Despite the higher potency of tazemetostat in biochemical assays, its effects on the viability of the tested cell lines were comparable with those of our two inhibitors, also when used in combination with temozolomide.

### MC4040 and MC4041 arrest GBM cell cycle in G0/G1 phase without apoptosis induction

In further investigation, we decided to better define the mechanism at the basis of GBM cell proliferation arrest by MC4040 and MC4041. We started by checking whether these EZH2 inhibitors induced apoptosis, through the evaluation of poly ADP-ribose polymerase 1 (PARP-1) expression. As shown by western blot analysis, nor MC4040 neither MC4041 induced PARP-1 cleavage up to 120 h of treatment in GL1 cells (Fig. 7a). As a positive control, the treatment with staurosporine (ST), a strong inducer of apoptosis, determined typical PARP-1 cleavage in the same cell line. (Figure 7a).

**Fig. 7:** **a** Western blot of GL1 untreated (ctr) and treated for 72 or 120 h with 25 μM MC4040 and MC4041 and for 6 h with 5 μM staurosporine (ST) showing uncleaved and cleaved PARP-1 and actin. **b** Western blot of GL1 and U-87 untreated (ctr) and treated for 72 h with 25 μM MC4040 showing p21 and p27 levels. **c** Cell cycle analysis of untreated and treated cells

Once determined that MC4040 and MC4041 did not induce apoptosis, we analysed the effects of these compounds on two negative regulators of cell cycle, p21 and p27, which are cyclin-dependent kinase inhibitors. We found that the basal expression of both p21 and p27 was quite low in GL1 and U-87 cells, while both markers were significantly upregulated after MC4040 treatment (25 μM, 72 h) in both cell lines (Fig. 7b). Additionally, flow cytometry cell cycle analysis revealed an accumulation of U-87 and GL1 cells in the G0/G1 phase after treatment with MC4040 or MC4041 (25 μM, 72 h) (Fig. 7c). These results suggested that MC4040 and MC4041 arrest cell proliferation at the G0/G1 phase by increasing p21 and p27 levels and do not induce apoptosis. Our findings strengthen the existing literature evidences documenting a G0/G1 cell cycle arrest after EZH2 inhibition in GBM cells [10, 38].

### MC4040 and MC4041 impair GBM aggressive and invasive phenotype by blocking neo-vascularization processes and reverting the EMT

Afterwards, we investigated in depth the molecular effects of our described compounds on U-87 and/or GL1 cells, to determine whether they could affect GBM aggressiveness and invasiveness. GBM is characterized by a proangiogenic and proinflammatory microenvironment [5]. Typically, neoangiogenesis is supported by high levels of secreted vascular endothelial growth factor (VEGF) [39]. Together with its “classical” functions, VEGF is also increasing the number of infiltrative macrophages participating in the establishment of an immunosuppressive microenvironment through the release of inhibitory cytokines [40]. Moreover, it has been shown that in the blood vessels of high-grade GBM the VEGFR1 levels are higher when compared with lower grade gliomas [41]. Interestingly, VEGFR1 is expressed by endothelial cells during vessel formation and remodelling, but it does not have a relevant role in physiological angiogenesis in adults [42]. Accordingly, VEGFR1 signalling has been related to tumour growth, progression, and metastasis, being involved in apoptosis inhibition and chemoresistance induction [43, 44]. In time, the VEGF/VEGFR1 signalling cascade has been studied in GBM and it was proven an interesting target to hit. Hence, we questioned ourselves if our EZH2 inhibitors could indirectly hit also this important pathway. We determined the expression of VEGFR1 and VEGF in untreated and MC4040-treated U-87 cells, expressing detectable basal protein levels of VEGF and its receptor VEGFR1, and we found that MC4040 was able to strongly reduce the levels of both proteins (Fig. 8).

**Fig. 8:** Immunofluorescence for VEGFR1 and for VEGF in untreated (ctr) and MC4040-treated (25 μM) U87 cells (left panels) for 48 h. The densitometry of all cells from five random fields taken in three different experiments are presented in the graphic (right panel) with the mean ± SD ***p < 0.001

In parallel, the effect of MC4040 and MC4041 on epithelial to mesenchymal transition (EMT) was analysed determining, in GL1 and U87 cells, the levels of E-cadherin as epithelial marker, of N-cadherin as mesenchymal marker, and of matrix metalloproteinases (MMPs), specifically MMP2, MMP3, and MMP9, basally upregulated in GL1 and U87 cells, and usually highly expressed in the majority of aggressive tumours and responsible for tumour invasiveness [15]. In these assays, MC4040 and MC4041 upregulated E-cadherin and downregulated N-cadherin, thus reverting the EMT process (Fig. 9a). Furthermore, MC4040 and MC4041 treatment decreased the expression of all the tested MMPs in U-87 and GL1 cells (Fig. 9a). In order to quantify the final readout of the effect of MC4040 and MC4041 on GBM cell invasiveness, we performed a Matrigel invasion assay. In both U-87 and GL1 cell lines the basal rate of motility was very high. The treatment with MC4040 and MC4041 markedly attenuated this malignant attitude (Fig. 9b, c), reducing the invasion capacity up to 4-fold. Taken together, our results demonstrate that our EZH2 inhibitors played an important role in reducing the angiogenic and invasive phenotype of GBM cells.

**Fig. 9:** **a** Western blot of EMT and invasion related proteins: E-cadherin, N-cadherin, MMP-2, MMP-3, and MMP-9. MC4040 and MC4041 were used at 20 μM for 48 h. The densitometry quantitation is indicated for each band normalized for actin band. **b** Matrigel invasion assay of U-87 and GL1 cells untreated (ctr) and treated with 20 μM MC4040 or MC4041 for 48 h. **c** Migrated cells were counted in five random fields. Three independent experiments were performed, and the results are presented with the mean ± SD **p < 0.01

### MC4040 and MC4041 display anti-inflammatory effects in GBM cells

Several different cancer types, including GBM, benefit of a chronically active inflammatory microenvironment, providing the proliferative and mutational incentive, necessary to unable the tumour to uncontrolled development. Histone methylation has been reported to epigenetically control the innate and adaptive immune responses [45]. Recently, several studies demonstrated that EZH2 plays a key role in inflammatory and autoimmune disorders. More in detail, EZH2 was reported to regulate cell adhesion and migration, with possible implications in leukocyte migration and immune responses [46], in production of inflammatory cytokines in dental pulp cells [47] or in macrophages [48], in regulation of microglial inflammatory gene expression [49], and in adaptative resistance to tumour immunotherapy [50]. The present evidences surely depict an articulated scenario in which EZH2 is a main regulator of inflammatory and immune processes at various levels.

To evaluate if EZH2 inhibition in GBM could impact on inflammation, and to gain further insight into the molecular mechanism of MC4040 and MC4041, we investigated on the expression patterns of the main inflammatory and anti-inflammatory cytokines in U-87 and GL1 cells in untreated and in MC4040- and MC4041-treated samples. As expected, both U-87 and GL1 expressed basally high levels of the pro-inflammation cytokines TGF-β, TNF-α and IL-6, and very low levels of the anti-inflammatory cytokine IL-10 (Fig. 10). The treatment with either MC4040 or MC4041 determined a significant decrease of TGF-β, TNF-α, and IL-6 and a significant increase of IL-10 (Fig. 10). These data show that U-87 and GL1 cells have a strong pro-inflammatory phenotype, that could contribute to their aggressiveness and proliferation. Here we provided a first evidence on the possibility to attenuate this attitude by treatment with the EZH2 inhibitors MC4040 and MC4041.

**Fig. 10:** Western blot of U-87 and GL1 untreated (ctr) and treated with 20 μM MC4040 or MC4041 for 48 h for TGF-ß, TNF-α, IL-6, IL-10, and actin. The densitometry quantification is indicated for each band normalized for actin band

## Discussion

Several different factors still obstacle the development of a proper cure for GBM, that remains the most common and aggressive malignant primary brain tumour in adults. To date, the sole chemotherapeutic agent in use against GBM is the alkylating drug temozolomide. The standard GBM treatment consists of surgical resection of the tumour, followed by chemotherapy and concomitant radiotherapy [2]. It is worth to point out that the current available treatment is not a cure. Hence, there is an urgent need for alternative and/or complementary therapeutic strategies and targets to hit. The epigenetic mechanisms underlying GBM development and progression are being elucidated and clarified. The SAM-dependent histone methyltransferase EZH2 has been found upregulated in gliomas and correlated with an aggressive phenotype [10, 11], while its depletion by RNA interference resulted in anti-glioma effects [12]. Importantly, some known EZH2 inhibitors have been already tested against GBM models in vitro and in vivo, confirming the biological evidences assessing the relevance of EZH2 as target in this disorder [16]. Here, we report the effects on GBM, including primary GBM cell cultures, of two novel EZH2 inhibitors, MC4040 and MC4041, containing a *N*-phenylpyrrole core decorated with a cyclic amine (morpholine, MC4040, or piperidine, MC4041), often present in known EZH2i, and carrying the 2-pyridone moiety known to be crucial for the EZH2 inhibiting activity [51]. When tested against a human five-component PRC2 complex, MC4040 and MC4041 displayed single-digit micromolar IC_50_ values against EZH2-PRC2 with a 10-fold selectivity over EZH1-PRC2. Importantly, the two novel compounds proved to be selective for EZH2/EZH1 over a panel of SAM-dependent methyltransferases including DNMT1, G9a, and PRMT1, displaying no inhibition of these targets up to 200 μM. Molecular docking and MMGBSA calculations helped us to shed light on the differences in the binding mode of the two newly synthesized compounds, explaining also the difference in activity recorded in biochemical assays. The two novel compounds have been tested on the primary GBM cell cultures GL1, GL2, and GL3 as well as on the GBM cell line U-87, displaying a dose- and time-dependent reduction of cell viability, without significant effect on human normal dermal fibroblast (HF) primary culture proliferation. Interestingly, the effects of the two newly synthesized EZH2 inhibitors were comparable to those of the clinically studied inhibitor tazemetostat, tested at the same doses and times. The MC4040- and MC4041-mediated EZH2 inhibition in U-87 and GL1 cells was confirmed by the decrease of the H3K27me3 levels, basally increased in both cell lines. Additionally, the combination of EZH2 inhibition with the standard GBM chemotherapy (temozolomide) was tested. The combination yielded much stronger, but not additive, effects with a 60% reduction of cell viability after 72 h. We have also found that MC4040 and MC4041 impair GBM cell viability by arresting cell proliferation at the G0/G1 phase by increasing p21 and p27 levels without inducing apoptosis. Our findings are in agreement with the existing literature evidences, documenting a G0/G1 cell cycle arrest after EZH2 inhibition in GBM cells [10, 38]. Additionally, we validated EZH2 as a valuable target to attenuate GBM malignant and aggressive phenotype. Hence, MC4040 and MC4041 treatment in GBM cells reduced VEGFR1 and VEGF expression, upregulated E-cadherin and downregulated N-cadherin and MMPs, reverting the EMT process. Accordingly, in a Matrigel invasion assay, the treatment with MC4040 and MC4041 markedly attenuated GBM cells motility, reducing the invasion capacity up to 4 folds respect to untreated cells. Noteworthy, to the best of our knowledge, we have shown for the first time that EZH2 inhibition impairs the pro-inflammatory GBM phenotype, that usually sustains and strengthens tumour development and aggressiveness. Specifically, the treatment of U-87 and GL1 cells with MC4040 or MC4041 determined a significant decrease of all the three tested pro-inflammatory TGF-β, TNF-α, and IL-6, as well as a significant increase of the anti-inflammatory IL-10 cytokines expression. Currently, we are working to shed light on the precise mechanism through which EZH2 inhibition impairs GBM aggressiveness and how it can impact on tumour-mediated immunomodulation and inflammation. We wish that our findings will stimulate and motivate new researches in this field, clarifying the complex molecular pathways and mechanisms at the bases of EZH2-mediated effects in GBM.

## Conclusions

In conclusion, the present study describes the design and synthesis of two novel and selective EZH2 inhibitors able to reduce H3K27 methylation levels in U-87 and GL1 GBM cells. MC4040 and MC4041 dose- and time-dependently impaired GBM cell viability arresting the cell cycle in the G0/G1 phase and potentiated the effects of temozolomide. We proved that EZH2 inhibition by MC4040 and MC4041 attenuates cancer malignant phenotype by reducing VEGFR1/VEGF expression, reverting the EMT process and inhibiting invasiveness. To the best of our knowledge, here, we show for the first time that targeting EZH2 in GBM displays anti-inflammatory effects, further strengthening the relevance of this target in this cancer type.

## Data Availability

All the published data are available. There is no supporting material.

## Abbreviations

AEBP2: Adipocyte enhancer-binding protein 2
BSA: Bovine serum albumin
DMEM: Dulbecco’s modified Eagle’s medium
DMF: *N*,*N*-Dimethylformamide DNMT1 DNA methyltransferase 1
DTT: Dithiothreitol
EDTA: Ethylenediaminetetraacetic acid
EED: Embryonic ectoderm development
EIMS: Electron ionization mass spectrometry
EMEM: Eagle’s minimum essential medium
EMT: Epithelial-mesenchymal transition
EZH1: Enhancer of zeste homologue 1
EZH2: Enhancer of zeste homologue 2
EZH2i: EZH2 inhibitors
FCS: Foetal calf serum
G9a (EHMT2): Euchromatic histone-lysine *N*-methyltransferase 2
GBM: Glioblastoma
GFAP: Glial fibrillary acidic protein
H3K27: Lysine 27 of the histone 3
H3K27me3: Trimethylated H3K27
HF: Human fibroblasts
IL: Interleukin
MB: Medulloblastoma
MDA-MB231: breast cancer cell line
MMGBSA: Molecular mechanics/generalized Born surface area
MMP: Matrix metalloproteinase
MT: Methyltransferase
NMR: Nuclear magnetic resonance
OD: Optical density
PARP: Poly ADP-ribose polymerase
PBS: Phosphate-buffered saline
PDB: Protein data bank
PMSF: Phenylmethanesulfonyl fluoride
PRC2: Polycomb repressive complex 2
PRMT1: Protein arginine methyltransferase 1
RbAp48: Retinoblastoma-associated protein 48
SAH: *S*-Adenosyl-L-homocysteine
SAM: *S*-Adenosyl-L-methionine
SDS: Sodium dodecyl sulphate
SHH: Sonic Hedgehog
ST: Staurosporine
SUZ12: Polycomb repressive complex 2 subunit
TAZ: Tazemetostat
TBTU: *O*-(Benzotriazole-1-yl)-*N*,*N*,*N'*,*N'*-tetramethyluronium tetrafluorborate
TGF-β: Transforming growth factor β
TLC: Thin layer chromatography
TMZ: Temozolomide
TNF-α: Tumour necrosis factor α
VEGF: Vascular endothelial growth factor
VEGFR1: Vascular endothelial growth factor receptor 1

## References

[1] Ostrom Quinn T., Gittleman Haley, Fulop Jordonna, Liu Max, Blanda Rachel, Kromer Courtney, Wolinsky Yingli, Kruchko Carol, Barnholtz-Sloan Jill S. (2015). CBTRUS Statistical Report: Primary Brain and Central Nervous System Tumors Diagnosed in the United States in 2008-2012. Neuro-Oncology.

[2] Wick W, Platten M (2018). Understanding and treating glioblastoma. Neurol Clin.

[3] Meyer M, Reimand J, Lan X, Head R, Zhu X, Kushida M, Bayani J, Pressey JC, Lionel AC, Clarke ID (2015). Single cell-derived clonal analysis of human glioblastoma links functional and genomic heterogeneity. Proc Natl Acad Sci U S A.

[4] Patel AP, Tirosh I, Trombetta JJ, Shalek AK, Gillespie SM, Wakimoto H, Cahill DP, Nahed BV, Curry WT, Martuza RL (2014). Single-cell RNA-seq highlights intratumoral heterogeneity in primary glioblastoma. Science.

[5] Buerki Robin A., Chheda Zinal S., Okada Hideho (2018). Immunotherapy of Primary Brain Tumors: Facts and Hopes. Clinical Cancer Research.

[6] Ferreira WA, Pinheiro Ddo R, Costa Junior CA, Rodrigues-Antunes S, Araujo MD, Leao Barros MB, Teixeira AC, Faro TA, Burbano RR, Oliveira EH (2016). An update on the epigenetics of glioblastomas. Epigenomics.

[7] Pangeni Rajendra P., Zhang Zhou, Alvarez Angel A., Wan Xuechao, Sastry Namratha, Lu Songjian, Shi Taiping, Huang Tianzhi, Lei Charles X., James C. David, Kessler John A., Brennan Cameron W., Nakano Ichiro, Lu Xinghua, Hu Bo, Zhang Wei, Cheng Shi-Yuan (2018). Genome-wide methylomic and transcriptomic analyses identify subtype-specific epigenetic signatures commonly dysregulated in glioma stem cells and glioblastoma. Epigenetics.

[8] Tan SK, Pastori C, Penas C, Komotar RJ, Ivan ME, Wahlestedt C, Ayad NG (2018). Serum long noncoding RNA HOTAIR as a novel diagnostic and prognostic biomarker in glioblastoma multiforme. Mol Cancer.

[9] Kim KH, Roberts CW (2016). Targeting EZH2 in cancer. Nat Med.

[10] Zhang J, Chen L, Han L, Shi Z, Zhang J, Pu P, Kang C (2015). EZH2 is a negative prognostic factor and exhibits pro-oncogenic activity in glioblastoma. Cancer Lett.

[11] Yin Y, Qiu S, Peng Y (2016). Functional roles of enhancer of zeste homolog 2 in gliomas. Gene.

[12] Suva ML, Riggi N, Janiszewska M, Radovanovic I, Provero P, Stehle JC, Baumer K, Le Bitoux MA, Marino D, Cironi L (2009). EZH2 is essential for glioblastoma cancer stem cell maintenance. Cancer Res.

[13] Fan TY, Wang H, Xiang P, Liu YW, Li HZ, Lei BX, Yu M, Qi ST (2014). Inhibition of EZH2 reverses chemotherapeutic drug TMZ chemosensitivity in glioblastoma. Int J Clin Exp Pathol.

[14] Fioravanti Rossella, Stazi Giulia, Zwergel Clemens, Valente Sergio, Mai Antonello (2018). Six Years (2012–2018) of Researches on Catalytic EZH2 Inhibitors: The Boom of the 2‐Pyridone Compounds. The Chemical Record.

[15] Yu T, Wang Y, Hu Q, Wu W, Wu Y, Wei W, Han D, You Y, Lin N, Liu N (2017). The EZH2 inhibitor GSK343 suppresses cancer stem-like phenotypes and reverses mesenchymal transition in glioma cells. Oncotarget.

[16] Grinshtein N, Rioseco CC, Marcellus R, Uehling D, Aman A, Lun X, Muto O, Podmore L, Lever J, Shen Y (2016). Small molecule epigenetic screen identifies novel EZH2 and HDAC inhibitors that target glioblastoma brain tumor-initiating cells. Oncotarget.

[17] Mellini Paolo, Marrocco Biagina, Borovika Diana, Polletta Lucia, Carnevale Ilaria, Saladini Serena, Stazi Giulia, Zwergel Clemens, Trapencieris Peteris, Ferretti Elisabetta, Tafani Marco, Valente Sergio, Mai Antonello (2018). Pyrazole-based inhibitors of enhancer of zeste homologue 2 induce apoptosis and autophagy in cancer cells. Philosophical Transactions of the Royal Society B: Biological Sciences.

[18] Miele E, Valente S, Alfano V, Silvano M, Mellini P, Borovika D, Marrocco B, Po A, Besharat ZM, Catanzaro G (2017). The histone methyltransferase EZH2 as a druggable target in SHH medulloblastoma cancer stem cells. Oncotarget.

[19] Joshi SD, Kumar D, More UA, Yang KS, Aminabhavi TM (2016). Design and development of pyrrole carbaldehyde: an effective pharmacophore for enoyl-ACP reductase. Med Chem Res.

[20] Yonekura K, Oki K, Tsuchimoto T (2016). Indium-Catalyzed Formal N-Arylation and N-Alkylation of Pyrroles with Amines. Adv Synth Catal.

[21] Verma SK, Tian X, LaFrance LV, Duquenne C, Suarez DP, Newlander KA, Romeril SP, Burgess JL, Grant SW, Brackley JA (2012). Identification of Potent, selective, cell-active inhibitors of the histone lysine methyltransferase EZH2. ACS Med Chem Lett.

[22] Berman H, Henrick K, Nakamura H (2003). Announcing the worldwide Protein Data Bank. Nat Struct Biol.

[23] Webb B, Sali A (2017). Protein structure modeling with MODELLER. Methods Mol Biol.

[24] Korb O, Stutzle T, Exner TE (2009). Empirical scoring functions for advanced protein-ligand docking with PLANTS. J Chem Inf Model.

[25] Jakalian A, Jack DB, Bayly CI (2002). Fast, efficient generation of high-quality atomic charges. AM1-BCC model: II. Parameterization and validation. J Comput Chem.

[26] Wang J, Wolf RM, Caldwell JW, Kollman PA, Case DA (2004). Development and testing of a general amber force field. J Comput Chem.

[27] Ramsey S, Nguyen C, Salomon-Ferrer R, Walker RC, Gilson MK, Kurtzman T (2016). Solvation thermodynamic mapping of molecular surfaces in AmberTools: GIST. J Comput Chem.

[28] Sousa da Silva AW, Vranken WF (2012). ACPYPE - AnteChamber PYthon Parser interfacE. BMC Res Notes.

[29] Izadi S, Anandakrishnan R, Onufriev AV (2014). Building water models: a different approach. J Phys Chem Lett.

[30] Maier JA, Martinez C, Kasavajhala K, Wickstrom L, Hauser KE, Simmerling C (2015). ff14SB: improving the accuracy of protein side chain and backbone parameters from ff99SB. J Chem Theory Comput.

[31] Genheden S, Ryde U (2015). The MM/PBSA and MM/GBSA methods to estimate ligand-binding affinities. Expert Opin Drug Discov.

[32] O'Boyle NM, Banck M, James CA, Morley C, Vandermeersch T, Hutchison GR (2011). Open Babel: An open chemical toolbox. J Cheminform.

[33] Halgren TA (1999). MMFF VI. MMFF94s option for energy minimization studies. J Comput Chem.

[34] Bianchi E, Taurone S, Bardella L, Signore A, Pompili E, Sessa V, Chiappetta C, Fumagalli L, Di Gioia C, Pastore FS (2015). Involvement of pro-inflammatory cytokines and growth factors in the pathogenesis of Dupuytren’s contracture: a novel target for a possible future therapeutic strategy?. Clin Sci (Lond).

[35] Hartwig JF, Kawatsura M, Hauck SI, Shaughnessy KH, Alcazar-Roman LM (1999). Room-temperature palladium-catalyzed amination of aryl bromides and chlorides and extended Scope of aromatic C-N bond formation with a commercial ligand. J Org Chem.

[36] Sabatino M, Rotili D, Patsilinakos A, Forgione M, Tomaselli D, Alby F, Arimondo PB, Mai A, Ragno R (2018). Disruptor of telomeric silencing 1-like (DOT1L): disclosing a new class of non-nucleoside inhibitors by means of ligand-based and structure-based approaches. J Comput Aided Mol Des.

[37] Miller BR, McGee TD, Swails JM, Homeyer N, Gohlke H, Roitberg AE (2012). MMPBSA.py: an efficient program for end-state free energy calculations. J Chem Theory Comput.

[38] Qi W, Chan H, Teng L, Li L, Chuai S, Zhang R, Zeng J, Li M, Fan H, Lin Y (2012). Selective inhibition of Ezh2 by a small molecule inhibitor blocks tumor cells proliferation. Proc Natl Acad Sci U S A.

[39] Dubois LG, Campanati L, Righy C, D’Andrea-Meira I, Spohr TC, Porto-Carreiro I, Pereira CM, Balca-Silva J, Kahn SA, DosSantos MF (2014). Gliomas and the vascular fragility of the blood brain barrier. Front Cell Neurosci.

[40] Lohr J, Ratliff T, Huppertz A, Ge Y, Dictus C, Ahmadi R, Grau S, Hiraoka N, Eckstein V, Ecker RC (2011). Effector T-cell infiltration positively impacts survival of glioblastoma patients and is impaired by tumor-derived TGF-beta. Clin Cancer Res.

[41] Baumgarten P, Blank AE, Franz K, Hattingen E, Dunst M, Zeiner P, Hoffmann K, Bahr O, Mader L, Goeppert B (2016). Differential expression of vascular endothelial growth factor A, its receptors VEGFR-1, -2, and -3 and co-receptors neuropilin-1 and -2 does not predict bevacizumab response in human astrocytomas. Neuro-Oncology.

[42] Roskoski R (2008). VEGF receptor protein-tyrosine kinases: structure and regulation. Biochem Biophys Res Commun.

[43] Fischer C, Mazzone M, Jonckx B, Carmeliet P (2008). FLT1 and its ligands VEGFB and PlGF: drug targets for anti-angiogenic therapy?. Nat Rev Cancer.

[44] Atzori MG, Tentori L, Ruffini F, Ceci C, Lisi L, Bonanno E, Scimeca M, Eskilsson E, Daubon T, Miletic H (2017). The anti-vascular endothelial growth factor receptor-1 monoclonal antibody D16F7 inhibits invasiveness of human glioblastoma and glioblastoma stem cells. J Exp Clin Cancer Res.

[45] Stender JD, Glass CK (2013). Epigenomic control of the innate immune response. Curr Opin Pharmacol.

[46] Gunawan M, Venkatesan N, Loh JT, Wong JF, Berger H, Neo WH, Li LY, La Win MK, Yau YH, Guo T (2015). The methyltransferase Ezh2 controls cell adhesion and migration through direct methylation of the extranuclear regulatory protein talin. Nat Immunol.

[47] Hui T, A P, Zhao Y, Wang C, Gao B, Zhang P, Wang J, Zhou X, Ye L (2014). EZH2, a potential regulator of dental pulp inflammation and regeneration. J Endod.

[48] Zhang W, Liu H, Liu W, Liu Y, Xu J (2015). Polycomb-mediated loss of microRNA let-7c determines inflammatory macrophage polarization via PAK1-dependent NF-kappaB pathway. Cell Death Differ.

[49] Arifuzzaman S, Das A, Kim SH, Yoon T, Lee YS, Jung KH, Chai YG (2017). Selective inhibition of EZH2 by a small molecule inhibitor regulates microglial gene expression essential for inflammation. Biochem Pharmacol.

[50] Zingg D, Arenas-Ramirez N, Sahin D, Rosalia RA, Antunes AT, Haeusel J, Sommer L, Boyman O (2017). The histone methyltransferase Ezh2 controls mechanisms of adaptive resistance to tumor immunotherapy. Cell Rep.

[51] Brooun A, Gajiwala KS, Deng YL, Liu W, Bolanos B, Bingham P, He YA, Diehl W, Grable N, Kung PP (2016). Polycomb repressive complex 2 structure with inhibitor reveals a mechanism of activation and drug resistance. Nat Commun.

